RETRACTED

# A Study on the Relationship between Sense of Disease Uncertainty and Family Strength and Mental Resilience in Guardians of Children with Inflammatory Bowel Disease

**DOI:** 10.1155/2022/4797281

**Published:** 2022-10-12

**Authors:** Jun Yan, Lin Luo

**Affiliations:** ^1^Wuhan Children's Hospital (Wuhan Maternal and Child Healthcare Hospital), Tongji Medical College, Huazhong University of Science&Technology, Wuhan 430014, China; ^2^ICU, Fifth Hospital in Wuhan, Wuhan 430050, China

## Abstract

**Background:**

Inflammatory bowel disease is difficult to cure, which seriously affects the physical and mental health of children and brings negative psychological stress to guardians. Uncertainty in illness of guardians reduces the ability of care and is not conducive to the treatment and recovery of children. Therefore, it is of great significance to explore the related factors of uncertainty in illness.

**Objective:**

The aim of this study is to explore the relationship between sense of disease uncertainty and family strength and mental resilience in guardians of children with inflammatory bowel disease (IBD).

**Method:**

A total of 146 guardians of 88 children with inflammatory bowel disease were investigated. The guardians' sense of disease uncertainty, family strength, and mental resilience were evaluated by Mishel uncertainty in illness scale-family member (MUIS-FM), family hardiness index (FHI), and Connor–Davidson resilience sca1e (CD-RISC), respectively. Spearman correlation was used for analyzing the correlation between the guardian's sense of disease uncertainty and family resilience.

**Results:**

The guardian's MUIS-FM score from lowest to highest was complexity, unpredictability, lack of information, and uncertainty. The average scores of FHI and CD-RISC were lower than the average score of CD-RISC of the general community in China 65.4 (*t* = −4.36, *P* < 0.05). The score of MUIS-FM was significantly correlated with the scores of FHI and CD-RISC (*P* < 0.05). Multiple linear regression analysis showed that the challenge score in the FHI scale and the fortitude score and the strength score in the CD-RISC scale were the main influencing factors of guardians' sense of disease uncertainty in children with IBD (*P* < 0.05).

**Conclusion:**

The guardians of children with IBD had a more serious sense of disease uncertainty, which was related to family strength and mental resilience.

## 1. Introduction

Inflammatory bowel disease (IBD) is a type of chronic nonspecific inflammation of the intestine with unknown etiology [1, 2]. It mainly includes Crohn's disease (CD) and ulcerative colitis (UC), which is often manifested as abdominal pain, diarrhea, bloody stools, weight loss, and so on. The disease is difficult to cure and has repeated attacks, with potential cancer risk. In recent years, the incidence of IBD among children has been increasing. IBD seriously affects growth, development, physiological function, and mental healthof children [3, 4]. Moreover, it is also a heavy negative stress event and psychological impact on the guardians, which leads to a series of psychological problems of the guardians, which has attracted more and more social attention [5, 6]. The psychological problems of guardians are often related to the family members' low understanding and awareness of the specific condition, treatment process, and prognosis of IBD. Uncertainty in illness refers to the lack of ability to determine disease information, including the etiology, pathogenesis, treatment plan, nursing measures, and prognosis of the disease, which is one of the main factors causing psychological pressure on patients or guardians and may lead to the weakening of guardians' ability to seek disease information. It is easy to cause a large number of adverse psychological states and extreme behaviors if guardians are prevented from playing their normal care-giving functions [7]. The uncertainty of the disease will adversely affect the normal living status and quality of life of the guardian, thus damaging the mental health of the guardian and is not conducive to the treatment and rehabilitation of the children [8]. Therefore, it is of great clinical significance to pay attention to the sense of disease uncertainty of guardians of children with IBD. Current studies on family members' sense of disease uncertainty mainly focused on comprehensive clinical specialties such as internal medicine, surgery, and oncology [9], while there were few reports on guardians of IBD children. This study mainly studied the correlation between the guardian's sense of disease uncertainty and family strength and mental resilience in children with IBD. The report was as follows.

RETRACTED

## 2. Materials and Methods

### 2.1. General Data

A total of 146 guardians of 88 children with inflammatory bowel disease were investigated. This study was approved by the Wuhan Children's Hospital (Wuhan Maternal and Child Healthcare Hospital) Ethics Committee. Children inclusion criteria were (1) the children were diagnosed as IBD according to the expert consensus on diagnosis and treatment of IBD in children in 2019 [10]; (2) 1–14 years old; (3) diseases were controlled during follow-up; (4) complete follow-up data. Exclusion criteria were (1) complicated with diabetes, cardiovascular and cerebrovascular diseases, liver and spleen dysfunction, infectious diseases, blood, or immune system diseases; (2) have taken drugs that affect platelets within two weeks, such as ticlopidine, heparin aspirin, and dipyridamole. There were 47 cases of CD and 41 cases of UC in the children. There were 56 males and 32 females. The onset age was (9.25 ± 2.41) years.

Guardian inclusion criteria were (1) age 18–70; (2) the education level was junior high school or above; (3) be the immediate relative of the child and the main caregiver and understand the general situation of the child; (4) in good health and to be able to complete the relevant evaluation of this study normally. Exclusion criteria were (1) the presence of serious physical diseases or mental disorders. A total of 146 guardians were aged from 26 to 66, with an average of (45.23 ± 13.15) years.

### 2.2. Evaluative Methods

During the outpatient visit or hospitalization, the guardian was evaluated with scales. One gastroenterology nurse was assigned to administer the scales. Before the test, the guardian should be explained to the purpose and basic methods of the test. Unified instructions were used for each scale, and the contents of the test that the guardian does not fully understand could be further analyzed. After the guardian fully understands the measurement content, the guardian would independently complete the evaluation of all scales according to their own actual situation, and the evaluation time was 30 min. The form would be returned on the spot after being filled in by the guardian. A total of 146 scales were issued, and 146 were recovered with a recovery rate of 100%. The method flow chart of this study is shown in Figure 1.

### 2.3. Assessment Content and Tools

Sense of disease uncertainty: the Chinese version of the scale Mishel uncertainty in illness scale-family member (MUIS-FM) [11] was used for evaluation, which was applied to measure the status of the guardian's sense of disease uncertainty. The content of the scale included 4 dimensions such as complexity, uncertainty, unpredictability, and lack of information. It included 33 items in total. The lowest score was 33 points, and the highest score was 165 points. The higher the score was, the stronger the uncertainty of the disease was. Dimension scores = (average score of dimension/highest score of dimension) × 100%.

Family strength: the family hardiness index (FHI) [12] was used for evaluating the internal strengths of family members. The scale included three dimensions of commitment, challenge, and control, with a total of 20 items. The Likert 4-level scoring method was adopted. A score of 1 was assessed as strongly disagree. A score of 2 was assessed as disagree. A score of 3 was assessed as agree. A score of 4 was assessed as strongly agree. Reverse scoring questions included the items 1, 2, 3, 8, 10, 14, 16, 19, and 20, and the remaining items were positive scoring questions. The higher the total score was, the better the family resilience was. Cronbach's coefficient of this scale was 0.80.

RETRACTED

Mental resilience: assessed by the Connor–Davidson resilience scale(CD-RISC) [13], jointly developed by Connor KM and Davidson JR, it contained 25 items in total. Domestic scholar Liu et al. [14] introduced and sinicized it, including three dimensions of tenacity, strength, and optimism. The total score was the sum of the scores of all items. Cronbach's coefficient and retest validity of the scale were 0.89 and 0.87, respectively, which were used to measure the positive psychological characteristics conducive to the individual's adaptation to adversity such as disease and adverse events. The 4-level scoring method was adopted, and the total score was 0–100. The higher the cumulative score of each item, the better the mental resilience.

### 2.4. Statistical Methods

SPSS 21.0 was used for statistical analysis of all data. The measurement data conforming to normal distribution was represented by the mean ± standard deviation, the measurement data not conforming to normal distribution was represented by the median (P25, P75), count data were represented by the number of cases or percentage, and correlation was the Spearman correlation analysis method. The test level was bilateral *α* = 0.05.

## 3. Results

### 3.1. General Information of the Guardian

In the general information of 146 guardians, female (52.74%), 45–59 years old (43.15%), college education or above (62.33%), unemployed or retired (58.90%), full understanding of the disease (49.32%), mother of the child (35.62%), and family monthly income 2001–3000 (43.15%) accounted for a high proportion, as shown in Table 1.

### 3.2. Guardian's MUIS-FM Rating

The MUIS-FM scores of 146 guardians in this study ranged from low to high in order of complexity, unpredictability, lack of information, and uncertainty, as shown in Table 2.

### 3.3. Guardian's FHI Rating

FHI averaged an overall score of 42.68, as shown in Table 3.

### 3.4. Guardian's CD-RISC Rating

The average score of CD-RISC was 61.55, lower than the average score of CD-RISC of the general community in China 65.4 (*t* = -4.36, *P* < 0.05), as shown in Table 4.

### 3.5. Correlation of the Guardian's MUIS-FM Score with the FHI Score and CD-RISC Score

The total score of MUIS-FM was significantly correlated with the total score of FHI and its dimensions, and the total score of MUIS-FM was significantly correlated with the total score of CD-RISC and its dimensions, as shown in Table 5.

RETRACTED

### 3.6. Multiple Linear Regression of Factors Influencing Guardian's Sense of Disease Uncertainty in Children with IBD Analysis Results (*n* = 130)

Multiple linear regression analysis was conducted with the total score of sense of disease uncertainty as the dependent variable and general information, family resilience, and psychological resilience as independent variables. The results showed that the challenge score in the FHI scale and the fortitude score and the strength score in the CD-RISC scale were the main influencing factors of guardians' sense of disease uncertainty in children with IBD (*P* < 0.05). The results of multiple linear regression analysis are shown in Table 6.

## 4. Discussion

According to the data analysis of this study, the MUIS-FM score of the guardians of IBD in children was higher than the domestic norm (*P* < 0.05), indicating that the guardians of IBD in children had a strong sense of disease uncertainty and lacked the ability to determine the etiology, pathogenesis, treatment plan, nursing measures, prognosis, and other information of IBD. This result was similar to that of Kang et al. [9]. According to relevant literature [9], guardians of children with IBD were uncertain about the diagnosis, symptoms, treatment, and prognosis of the disease. It was concluded that guardians' cognition was mainly affected by the following four factors: (1) the symptoms of the disease were not clear; (2) lack of information and knowledge about disease diagnosis; (3) complex nursing and treatment; (4) the disease process and prognosis were unpredictable. In this study, the average total score of guardian uncertainty was 89.32, which was in the middle level. Through the observation of the scores of each dimension, the highest score index was uncertainty, while the lowest score was complexity, which indicated that the guardian disease of inflammatory bowel disease in children had a sense of uncertainty on the change of illness, prognosis, and treatment measures [8, 15]. Inflammatory bowel disease (IBD) was a chronic nonspecific inflammation of the intestine, characterized by repeated attacks and difficult radical cure, and had the risk of cancer [16]. In addition, the disease would cause abdominal pain, diarrhea, bloody stools, weight loss and other symptoms, causing malnutrition, fever, conjunctivitis, arthritis, and other systemic reactions. If complications occur in children, the condition of IBD will be rapidly aggravated, affecting the recovery of the disease, which is not conducive to the prediction of IBD. At the same time, the aggravation of the illness will cause the guardian to worry and cause anxiety and other negative emotions, resulting in a sense of disease uncertainty [17]. Since the treatment period of IBD was long and there were many adverse reactions of drugs (such as purine preparations and glucocorticoids), the guardian was concerned that the adverse reactions of drugs would affect the normal growth and development of the children and make the guardian feel uncertain about the treatment of the disease. In addition, it was a common phenomenon that children's drug tolerance and compliance were reduced in the treatment process. Parents did not understand this and mistakenly believed that the treatment was ineffective or aggravated the condition, which would further aggravate the uncertainty of the disease and affected the disease control and treatment [18]. In this study, most parents came from rural areas with a low education level, limited access to disease information and ability, and lack of disease treatment and nursing knowledge, resulting in a sense of uncertainty [19].

RETRACTED

Correlation analysis of this study showed that the MUIS-FM score was negatively correlated with the FHI total score and MUIS-FM dimensions (commitment, control, challenge) and the CD-RISC total score and CD-RISC dimensions (tenacity, strength, optimism) (*P* < 0.05), and multiple linear regression analysis showed that the challenge score in the FHI scale and the fortitude score and the strength score in the CD-RISC scale were the main influencing factors of guardian disease uncertainty in children with IBD. It was suggested that the stronger the guardian's disease uncertainty was, the weaker the family challenge ability was and the lower the psychological fortitude and strength were; on the contrary, the weaker the guardian's disease uncertainty was, the stronger the family challenge ability and the guardian's psychological fortitude and strength were, which was consistent with the relevant research results. Family resilience refers to the family characteristics and attributes that family members use internal resources to adapt to the stressful environment and successfully overcome the crisis under pressure. The challenge dimension is one of the key components of family resilience. Studies had shown that family resilience had a protective effect on families [20, 21]. Therefore, when the guardian faced the long-term ill children in repeated treatment, the psycology of guardians would have a strong sense of crisis and be severely hit. This situation may cause family instability, especially for families with poor family resilience [22].

The guardian could not correctly view the disease of the children, and there were phenomena such as mutual shirking of responsibility, distrust, and disagreement among family members. The lack of family's ability to challenge the disease affected the treatment of the children, resulting in a high sense of uncertainty about the disease. Mental resilience was the ability to rebound in the face of difficulties and setbacks. When the mental resilience of guardians was poor, their psychological and coping ability, tenacity, and stress resistance would also be reduced, and they were unwilling to face a series of pains brought by the disease and adopted negative coping methods so that their disease uncertainty would increase [23, 24]. Nursing staff should give guardians of children with disease-related knowledge education, improve the confidence of cure, improve the level of mental resilience, and reduce the sense of uncertainty of disease.

RETRACTED

## 5. Strengths and Limitations

The significance of this study was that the results shown that the illness uncertainty of the guardians of children with inflammatory bowel disease was more serious, which was related to the resilience and psychological resilience of their families. This conclusion suggested that there was a strong sense of illness uncertainty in the guardians of children with inflammatory bowel disease, and attention to the overall family harmony and psychological tolerance of the guardians of children with inflammatory bowel disease should not be ignored. Therefore, this study had certain guiding significance for the treatment of children with inflammatory bowel disease. However, the small number of subjects included in this study may lead to bias in the study results. Therefore, future studies should increase the sample size to further verify the results of this study.

## 6. Conclusions

In conclusion, the guardians of children with IBD had a more serious sense of disease uncertainty, which was related to family resilience and psychological resilience. The guardians of inflammatory bowel disease in children had a strong sense of disease uncertainty, so it was important to pay attention to the overall family harmony and psychological tolerance of the guardians of IBD in children.

## Figures and Tables

**Figure 1:** Method flow chart. IBD: inflammatory bowel disease, MUIS-FM: Mishel uncertainty in illness scale-family member, FHI: family hardiness index, CD-RISC: Connor–Davidson resilience scale. A total of 146 guardians of children with inflammatory bowel disease were investigated. The guardians' sense of disease uncertainty, family strength, and mental resilience were evaluated by MUIS-FM, FHI, and CD-RISC, respectively. These analyzed the correlation of MUIS-FM between FHI and CD-RISC, and the influencing factors of uncertainty in illness were analysed by multiple linear regression.

RETRACTED

**Table 1:** General information of the guardian.

Items	Number of people	Percentage
Gender		
Male	69	47.26
Female	77	52.74
Age (years)		
<45	51	34.93
45–59	63	43.15
≥60	32	21.92
Marital status		
Married	126	86.30
Unmarried, divorced, or widowed	20	13.70
Schooling		
Junior and senior secondary	55	37.67
College degree or above	91	62.33
Employment status		
Be on the job	60	41.10
Unemployed or retired	86	58.90
Knowledge of the disease		
Know thoroughly	72	49.32
Know	69	47.26
Know nothing	5	3.42
Relationship with children		
Father	48	32.88
Mother	52	35.62
Grandfather	12	8.22
Grandmother	13	8.90
Maternal grandfather	12	8.22
Maternal grandmother	9	6.16
Average monthly family income (yuan)		
<1000	8	5.48
1000–2000	51	34.93
2001–3000	63	43.15
>3000	24	16.44

**Table 2:** Guardian's MUIS-FM rating.

Items	Number of entries	Divide entries	Dimension scores	Average Score	Score ranges	Score index (%)
Unpredictability	5	3.43 (3,3.8)	17 (15,2)	17.17	6–25	68.68
Lack of information	7	3.27 (2.9,3.6)	23 (20,3)	22.86	13–32	71.44
Complexity	13	1.39 (1.2,1.5)	18 (16,2)	18.04	13–29	62.21
Uncertainty	8	3.88 (3.3,4.5)	31 (26,36)	31.24	13–40	78.10
Total points	33	2.7 (2.6,2.9)	89.5 (84,95)	89.32	66–112	79.75

**Table 3:** Guardian's FHI rating.

Items	Number of entries	Divide entries	Dimension scores	Average Score	Score ranges
Commitment	9	2.1 (1.9,2.3)	19 (17,2)	19.15	9–27
Control	6	2.0 (1.7,2.3)	12 (10,14)	12.34	6–21
Commitment	5	2.2 (1.8,2.6)	11 (9,13)	11.19	5–20
Total points	20	2.2 (1.9,2.3)	43 (38.75,46)	42.68	27–59

**Table 4:** Guardian's CD-RISC rating.

Items	Number of entries	Divide entries	Dimension scores	Average Score	Score ranges
Tenacity	13	2.3 (1.9,2.6)	30 (25,34.3)	30.12	12–50
Strength	8	2.6 (2.1,3.2)	21 (17,25.3)	21.03	8–32
Optimism	4	2.6 (2,3.3)	10.5 (8,13)	10.40	1–16
Total points	25	2.4 (2.2,2.7)	61 (54,68)	61.55	41–87

**Table 5:** Correlation of the guardian's MUIS-FM score with the FHI score and CD-RISC score.

Items		FHI				CD-RISC			
		Commitment	Control	Commitment	Total points	Tenacity	Strength	Optimism	Total points
MUIS-FM	*r*	−0.276	−0.230	−0.406	−0.462	−0.433	−0.438	−0.325	−0.386
	*P*	0.001	0.005	<0.001	<0.001	<0.001	<0.001	<0.001	0.027

**Table 6:** Multiple linear regression of factors influencing the guardian's sense of disease uncertainty in children with IBD analysis results.

Items	*B*	*SE*	*β*	*t*	*P*
Constant	123.676	4.822	—	25.650	<0.001
Commitment	−0.186	0.190	−0.074	−0.977	0.330
Control	−0.213	0.207	−0.075	−1.029	0.305
Commitment	−0.570	0.200	−0.211	−2.855	0.005
Tenacity	−0.324	0.086	−0.279	−3.772	<0.001
Strength	−0.367	0.115	−0.234	−3.191	0.002
Optimism	−0.240	0.216	−0.086	−1.109	0.269
Average monthly family income	0.000	0.001	−0.073	−1.043	0.299

RETRACTED

## Data Availability

The data used for this study have been included within the manuscript.

## References

[1] Seyedian S. S., Nokhostin F., Malamir M. D. (2019). A review of the diagnosis, prevention, and treatment methods of inflammatory bowel disease. *Journal of Medicine and Life*.

[2] Guan Q. (2019). A comprehensive review and update on the pathogenesis of inflammatory bowel disease. *Journal of Immunology Research*.

[3] Aardoom M. A., Veereman G., de Ridder L. (2019). A review on the use of anti-TNF in children and adolescents with inflammatory bowel disease. *International Journal of Molecular Sciences*.

[4] van Rheenen P. F. (2021). Managing abnormal liver tests in children with inflammatory bowel disease. *Current Opinion in Pediatrics*.

[5] Michel H. K., Siripong N., Noll R. B., Kim S. C. (2020). Caregiver and adolescent patient perspectives on comprehensive care for inflammatory bowel diseases: building a family-centered care delivery model. *Crohn’s & colitis 360*.

[6] Yue A., Pu X., Zheng W., Wang B., Yang Z., Shi Y. (2022). Relation of social-emotional development of infants to depressive symptom and positive parenting behavior of caregivers in poor rural areas. *Chinese Mental Health Journal*.

[7] Han Z. T., Zhang H. M., Wang Y. M., Zhu S. S., Wang D. Y. (2021). Uncertainty in illness and coping styles: moderating and mediating effects of resilience in stroke patients. *World Journal of Clinical Cases*.

[8] Arias-Rojas M., Carreño-Moreno S., Posada-López C. (2019). Uncertainty in illness in family caregivers of palliative care patients and associated factors. *Revista Latino-Americana De Enfermagem*.

[9] Kang J., Cho Y. J., Choi S. (2020). State anxiety, uncertainty in illness, and needs of family members of critically ill patients and their experiences with family-centered multidisciplinary rounds: a mixed model study. *PLoS One*.

[10] Ricciuto A, Aardoom M., Orlanski-Meyer E. (2021). Predicting outcomes in pediatric crohn’s disease for management optimization: systematic review and consensus statements from the pediatric inflammatory bowel disease–ahead program. *Gastroenterology*.

[11] Verduzco-Aguirre H. C., Babu D., Mohile S. G. (2021). Associations of uncertainty with psychological health and quality of life in older adults with advanced cancer. *Journal of Pain and Symptom Management*.

[12] Peng Y., Wang J., Sun G., Liu S. (2021). Family hardiness in patients with heart failure: exploring protective factors and identifying the mediator. *Psychology Research and Behavior Management*.

[13] Velickovic K., Rahm Hallberg I., Axelsson U. (2020). Psychometric properties of the connor-davidson resilience scale (CD-RISC) in a non-clinical population in Sweden. *Health and Quality of Life Outcomes*.

RETRACTED

[14] Liu X., Liu C., Zhao J., Li W., Li W., Zheng R. (2022). Reliability and validity of the 10-item resilience sale in Chinese community-dwelling adults. *Chinese Journal of Behavioral Medicine and Brain Science*.

[15] Lan C. F., Nie C. L., Lin Y. J. (2021). Uncertainty in illness and the coping styles of severe patients with COVID-19: current status and correlation. *Epidemiology and Infection*.

[16] Nielsen O. H., Gubatan J. M., Juhl C. B., Streett S. E., Maxwell C. (2022). Biologics for inflammatory bowel disease and their safety in pregnancy: a systematic review and meta-analysis. *Clinical Gastroenterology and Hepatology*.

[17] Guan T., Qan’ir Y., Song L. (2021). Systematic review of illness uncertainty management interventions for cancer patients and their family caregivers. *Supportive Care in Cancer*.

[18] Feingold J. H., Kaye-Kauderer H., Mendiolaza M., Dubinsky M. C., Keefer L., Gorbenko K. (2021). Empowered transitions: understanding the experience of transitioning from pediatric to adult care among adolescents with inflammatory bowel disease and their parents using photovoice. *Journal of Psychosomatic Research*.

[19] D’Agostino McGowan L., Grantz K. H., Murray E. (2021). Quantifying uncertainty in mechanistic models of infectious disease. *American Journal of Epidemiology*.

[20] Ruiz B. O., Zerbetto S. R., Galera S. A. F., Barcellos Fontanella B. J., Gonçalves A. M. D. S., Protti-Zanatta S. T. (2021). Family resilience: perception of family members of psychoactive substance dependents. *Revista Latino-Americana de Enfermagem*.

[21] Dunst C. J. (2021). Family hardiness and parent and family functioning in households with children experiencing adverse life conditions: a meta-analysis. *International Journal of Psychology Research*.

[22] Li S., Lin Z., Bian Q., Wang M., Lin L., Zhang H. (2017). Research on resilience and family hardiness of patients with Inflammatory Bowel Disease. *Chinese Nursing Management*.

[23] Toledano-Toledano F., Luna D., Moral de la Rubia J. (2021). Psychosocial factors predicting resilience in family caregivers of children with cancer: a cross-sectional study. *International Journal of Environmental Research and Public Health*.

[24] Kukihara H., Yamawaki N., Ando M., Nishio M., Kimura H., Tamura Y. (2020). The mediating effect of resilience between family functioning and mental well-being in hemodialysis patients in Japan: a cross-sectional design. *Health and Quality of Life Outcomes*.

